The article "Application of Mathematical Methods Based on Improved Fuzzy Computing in Building and Urban Design in the Environment of Industry 4.0" was published in 2022. Journal: Comput Intell Neurosci.

# Application of Mathematical Methods Based on Improved Fuzzy Computing in Building and Urban Design in the Environment of Industry 4.0

**DOI:** 10.1155/2022/3449431

**Published:** 2022-05-27

**Authors:** Chuan Duan

**Affiliations:** School of Architecture and Civil Engineering, Xihua University, Chengdu 610039, China

## Abstract

In order to improve the performance of the urban building in urban design, this paper uses the mathematical method based on an improved fuzzy calculation to construct an intelligent building and urban design system. Moreover, this paper quantitatively studies the pedestrian wind environment of high-rise buildings and determines the optimal building aerodynamic shape and optimal building layout in the full wind direction. In addition, based on the results of the whole watershed analysis of CFD numerical simulation, this paper reveals the mechanism of building shape and layout in the pedestrian wind environment of high-rise buildings. Finally, this paper constructs an intelligent model to improve the effect of urban architectural design. Through the model research results, we can see that the urban design intelligent system proposed in this paper meets the needs of urban design in the environment of Industry 4.0.

## 1. Introduction

In the context of Industry 4.0, there are very few cases where the development of AI application science is supported by mainstream architects and urban designers. Early claims of artificial intelligence have raised concerns that the core jobs and competencies of architects and urban designers will be displaced. At the same time, when expectations fail to materialize, there is a loss of interest and funding for AI in building and urban design. However, interest in AI has picked up again since the second decade of the twenty-first century. Advances in technology, changing attitudes towards computer science in general, the emergence of big data and data analytics, the widespread use of civics, the rediscovery of civic design, the emergence of civic design science, and large-scale open online design approaches are working together to advance a more positive outlook for AI in building and urban design and may lead to compelling outcomes.

At present, the phenomenon of blindly copying foreign architectural creations is common in domestic building and urban design, which is obviously in mourning with the idea of a “harmonious society”. In response to this phenomenon, we believe that we should not only actively absorb the good parts of the foreign building in architectural creation. What is more important is to absorb the excellent ideas in the development of foreign cities, such as the idea of focusing on the coordinated development of individual buildings and the city as a whole, to consider the issue of architectural creation in the context of macro urban society. Therefore, in order to realize a “harmonious society”, it is necessary to emphasize the concept of coordination between people, buildings, and the environment in architectural creation.

The article "Application of Mathematical Methods Based on Improved Fuzzy Computing in Building and Urban Design in the Environment of Industry 4.0" was published in 2022. Journal: Comput Intell Neurosci.

The huge demand in the construction market and the relatively affluent social and economic conditions have led to the phenomenon of the one-sided pursuit of form and blind pursuit of novelty in the field of urban and architectural design. This “impetuous” design idea is reflected in the urban environment. First of all, various construction projects compete with each other to become the city's logo and image projects. It is conceivable that every building strives to highlight its individual image and play a leading role in the city. The result is a cluttered urban landscape and weakens the overall appearance of the city. In addition, driven by the concept of the supremacy of form, urban architectural design is seriously plagiarized, applying some avant-garde and trendy fashion designs in the world, ignoring the specific base environment and cultural connotation; this leads to the disappearance of the environmental identity and cultural identity of urban areas. Many traditional urban areas and historical areas have been completely “renovated” after renovation, cutting off the social life network of the original residents, and the architectural form has become a false stage setting. The root cause of these problems lies in the neglect of the relationship between the part and the whole in creative activities and the lack of respect for the urban environment and regional culture. This self-centered view of creation will inevitably bring chaos to the overall urban environment, which is not conducive to the construction of a “harmonious society”. Therefore, we should adhere to the people-oriented scientific development concept, deal with the relationship between architecture and the city from an overall perspective, and realize the harmonious development of people, buildings, and the environment.

From urban planning and design to architectural design, it is a “three-stage” relationship from the whole to the group and then to the individual [1]. If the individual building is taken out and analyzed again, the overall volume of the building, the volume transition relationship, and the detail processing will form a “three-stage” relationship [2]. In this way, when the building is enlarged into a system, the details of the near-human scale are at its most microscopic level. However, the building volume observed from the city's perspective becomes its macro scale, and it is observed from the perspective of the street, that is, urban design [3].

The article "Application of Mathematical Methods Based on Improved Fuzzy Computing in Building and Urban Design in the Environment of Industry 4.0" was published in 2022. Journal: Comput Intell Neurosci.

This paper combines the mathematical method of improving fuzzy calculation to construct the intelligent building and urban design system and improves the effect of urban architectural design through the intelligent model.

## 2. Related Work

The methods and capabilities of urban architectural planning and design continue to develop with the advancement of science and technology. In the early urban architectural planning, due to the use of traditional manual drawings for design, there were many problems due to the limitation of technology such as low labor efficiency, long design and design cycles of drawings, and error-prone architectural planning and design information. It is difficult to exchange and store design files and design results [4] and so on. The improvement of the economic level and the acceleration of the urbanization process affect the needs of urban architectural planning and design, and the traditional manual drawing method cannot handle a large number of design documents quickly and accurately. Information technology and CAD software have begun to be popularized on a large scale, various industries have also begun to enter the digital age, and the “electronic design” system of the urban architectural planning and design industry has emerged as the times require [5]. The electronic construction report design system adopts CAD electronic drawings in a unified and standardized format, which can quickly extract and calculate and analyze the information to be designed for the building, complete the automatic quantitative accounting of design indicators, realize electronic filing, and dynamically store architectural project design plans. The precise data processing capability of CAD provides efficient and accurate design technology for architectural planning, and the specification standards and accounting indicators formulated by electronic design make the design results reasonable and serious [6]. With the increasingly complex development of urban architecture, urban planning and design need more comprehensive and objective analysis, and the CAD technology based on a two-dimensional plane is difficult to realize the image description of urban three-dimensional geospatial information [7].

At the beginning of the twenty-first century, the rapid development of 3D GIS technology made the concept of the digital city begin to be valued by people. The 3D visualization analysis of the architectural space environment in the digital city has become the development direction of architectural planning and design [8]. 3D GIS technology can be used for urban architectural planning and design. Comprehensive, intuitive, and scientific decision analyses are provided. In recent years, the fusion technology of BIM and GIS has attracted much attention in many industries, and its application in urban architectural planning and design has also entered the stage of research and exploration. BIM technology is widely used in some developed countries abroad [9]. Professional architectural engineering software based on BIM technology includes Revit and Infraworks series software products of Autodesk Company of the United States, ArchiCAD software of Graphisoft Company of Hungary, and MicroStation TriForma software of Bentley Company [10]. These large software developers provide comprehensive solutions for the needs of different stages of construction projects and the management goals of different professions. However, at present, most of these softwares are aimed at single building projects, which have poor support for terrain data and limited data capacity, which cannot meet the needs of urban planning and design in a three-dimensional environment. On the other hand, geographic information system (GIS) software is also moving closer to BIM. The processing of spatial data is a feature of GIS [11], and the storage, expression, and analysis of large-scale terrain spatial data are the strength of GIS, which just makes up for the shortcomings of traditional BIM software in infrastructure construction projects in a large-scale environment [12]. BIM and GIS are different in the geometric and semantic expressions of model objects. The key to their integrated application lies in the fusion of model data. With the in-depth research on the integration of BIM and GIS technology, although relevant personnel of various majors has completed the exchange of information and data through simple model conversion, similar methods only save part of the semantic information, resulting in obvious limitations in the application of BIM [13]. At present, the research on BIM and GIS integration mainly focuses on two aspects, one is the integration of basic data models, and the other is the integration of existing data formats. The former analyzes the different expression types of BIM and GIS model objects and establishes a unified expression model for the two [14].

The article "Application of Mathematical Methods Based on Improved Fuzzy Computing in Building and Urban Design in the Environment of Industry 4.0" was published in 2022. Journal: Comput Intell Neurosci.

At this stage, most research directions are mainly focused on the latter, integrating model data in different formats, such as IFC Explorer developed by the Karlsruhe University of Technology in Germany, BIM Server developed by the Eindhoven University of Technology in the Netherlands, and Navisworks software developed by Autodesk [15]. Among them, IFCExplorer CityGML is committed to the seamless integration of the BIM standard model format IFC and the GIS standard model format CityGML, but it is difficult to achieve indiscriminate conversion between the two standard models, and it is still at the lower level of detail of the research model conversion [16]. BIMServer software supports the understanding and management of various BIM model structures, and at the same time, it can realize the simple conversion of BIM to GIS models. However, its functions are limited to data management and transformation and cannot achieve application analysis [17]. In addition, the conversion between its BIM and GIS models still has problems such as poor quality of the converted model and lack of semantics. Although Navisworks can realize the integrated analysis and application of BIM data sets, it is mainly based on a simple file system, so it is difficult to process large-scale data and the efficiency is low. And its support for GIS data can only be achieved through the conversion of third-party software, which will inevitably lose a lot of real information during the conversion process [18].

## 3. Architecture and Urban Design Based on Improved Fuzzy Computing

The structural model used in this paper is a single building with a square cross section. The scale ratio used in the numerical simulation is consistent with the experiment, which is 1 : 500, and the size after the scale is *D*_*x*_ × *D*_*y*_ × *D*_*z*_=0.1 × 0.1 × 0.8*m* (Figure 1(a)), and Figure 1(b) shows the distribution of measuring points around the building. All the measuring points are located at the pedestrian height, and a total of 280 measuring points are arranged. The distribution range of measuring points is X × Y=0.792 × 0.792 m (the center point of the building is the origin of coordinates), which is about 8 times the cross-sectional area of the calculated model. The height H of the building is taken as the reference height, and *U*_ref_=11.3m/s, *I*_*u*_=11.6% at the reference height. Existing research conclusions show that, for the fitting of regions with lower heights, the logarithmic wind profile is better than the exponential wind profile. Since this paper studies the pedestrian wind environment at the pedestrian height (the height is 2 meters), in order to ensure the accuracy of the numerical simulation, the logarithmic wind profile is used for calculation. The distribution map of the measuring points is shown in Figure 1(c).

### 3.1. Calculation Domain and Boundary Condition Setting

In the CFD numerical simulation, the dimensions of all models are consistent with the wind tunnel test, and the size of the three-dimensional computational domain is set to *D*_*x*_ × *D*_*y*_ × *D*_*z*_=15*H* × 10*H* × 6*H* (Figure 2). After calculation, the corresponding blocking rate is less than 3%, which meets the corresponding requirements.

The article "Application of Mathematical Methods Based on Improved Fuzzy Computing in Building and Urban Design in the Environment of Industry 4.0" was published in 2022. Journal: Comput Intell Neurosci.

The inlet of the computational domain is set to velocity inlet, the outlet is set to pressure outlet, and the boundary conditions on both sides and the top boundary are symmetric boundary conditions (symmetry).

The model is structured and meshed with ICEM CFD software. In meshing, because the Reynolds number of the fluid in the near-wall region is low during the flow process, in order to ensure the full development of turbulence, the mesh in the near-wall region must be refined. On the other hand, since different turbulence models have different requirements for mesh quality, it is necessary to divide meshes of different sizes according to the selected turbulence model.

In the CFD calculation, the size of the first layer grid of the model is often determined by calculating the size of the *y* + value. The relevant calculation steps are as follows.

(1) It calculates the Reynolds number *Re*
  (1) $$\begin{array}{c} R_{e}=\frac{\rho UL}{\mu }. \end{array}$$
(2) It calculates the wall friction coefficient C_f_
  (2) $$\begin{array}{c} C_{f}={\left(2\;\log_{10}R_{e}-0.65\right)}^{-2.3}\left(R_{e}\leq 10^{9}\right). \end{array}$$
(3) It calculates the wall shear stress *τ*_w_
  (3) $$\begin{array}{c} \tau_{w}=C_{f}\times \frac{1}{2}\rho U^{2}. \end{array}$$
(4) It calculates the grid height of the first layer

(4) $$\begin{array}{c} u^{*}=\sqrt{\frac{\tau_{w}}{\rho }},\\ \Delta y=\frac{y^{+}\;\mu }{\rho u^{*}}. \end{array}$$

When meshing, it is often necessary to divide different meshes according to different calculation models. In order to facilitate the calculation, this paper uniformly selects Y^+^=15 for mesh division, the corresponding first-layer mesh size is set to Δ*y*=0.0005*m* after calculation, and the corresponding mesh schematic diagram and calculation conditions are set as shown in Figure 3.

In order to verify the influence of the mesh size on the calculation results, the working condition RANS-1 is used as the reference condition to verify the influence of different mesh sizes on the calculation results. Two sets of grids with different sizes were established on the basis of the working condition SCRS-1. The minimum grid size of the refined grid is 0.0005 m, the minimum grid size of the sparse grid is 0.002 m, and other related settings remain unchanged. The corresponding mesh numbers are as follows. The total number of refined meshes is about 9 × 10^7^, and the number of sparse meshes is about 4 × 10^7^. The comparison chart of different size grids is shown in Figure 4.

The article "Application of Mathematical Methods Based on Improved Fuzzy Computing in Building and Urban Design in the Environment of Industry 4.0" was published in 2022. Journal: Comput Intell Neurosci.

In the numerical simulation study in the pedestrian wind environment, the accuracy of the simulation calculation cannot be guaranteed due to the low height of pedestrians, which are easily affected by the ground roughness. Therefore, one of the key issues of CFD numerical simulation is to meet the requirement of wind speed self-sustainability in the empty flow domain, that is, to ensure that the flow characteristics of the flow field remain consistent in the horizontal direction when the fluid passes the ground surface.

In the CFD calculation, we first calculate an airflow field before starting the model calculation, from which we obtain the average wind profile at the entrance, exit, and three locations of the model. The wind profile without corresponding adjustment is shown in Figure 5, and it can be found that the unadjusted wind profile does not achieve good retention at lower altitudes. At this altitude, the wind speed profile is significantly affected, resulting in a change in wind speed. In order to keep the wind speed uniform at lower heights, the self-sustainability of the wind speed is achieved by modifying the wall function and roughness parameters in this paper.

It can be found that in the wind field after debugging, the wind speeds of the inlet and outlet surfaces are consistent, thus ensuring the accuracy of the numerical simulation in this paper.

When evaluating the pedestrian wind environment around a building, the wind speed ratio *R*_*i*_ is often used for analysis, and its related definition is as follows:

(5) $$\begin{array}{c} R_{i}=\frac{V_{i}}{V_{0}}, \end{array}$$

where *V*_*i*_ is the wind speed at the pedestrian height at the measuring point around the building (this paper is 2 meters above the ground), and *V*_0_ is the wind speed at the entrance pedestrian height when there is no building [19].

In order to find the turbulence model with the best match between the predicted results and the experimental results, the turbulence model is judged by three evaluation indicators. The corresponding parameters are as follows:

(1) The indicator *q* is
  (6) $$\begin{array}{c} q=\frac{1}{M}\sum_{i=1}^{M}n_{i},\\ n_{i}=\left\{\begin{array}{c} 1\\ 0 \end{array}\left|\frac{R_{i\;\exp}-R_{iCF\;D}}{R_{i\;\exp}}\right|\leq 0.2\text{ or }\left|R_{i\;\exp}-R_{iCF\;D}\right|\leq 0.2\right.. \end{array}$$
(2) The average error *δ* is
  (7) $$\begin{array}{c} \delta =\frac{1}{M}\sum_{i=1}^{M}\left|R_{\text{iexp}}-R_{\text{iCFD}}\right|. \end{array}$$
(3) The mean square error *σ* is

(8) $$\begin{array}{c} \sigma =\sqrt{\frac{1}{M}\sum_{i=1}^{M}{\left(R_{\text{exp}}-R_{iCF\;D}\right)}^{2}}. \end{array}$$

In the above three formulas, *M* is the number of measuring points, and *R*_iexp_, *R*_*iCF*  *D*_ is the wind tunnel test result and CFD simulation result at the i-th measuring point, respectively.

The article "Application of Mathematical Methods Based on Improved Fuzzy Computing in Building and Urban Design in the Environment of Industry 4.0" was published in 2022. Journal: Comput Intell Neurosci.

After sorting out the wind tunnel test data, a total of 244 valid data measurement points are collected in the wind tunnel test. Through statistical analysis of these 244 different measuring points, it is found that there are 77 low wind speed measuring points (wind speed ratio *R*_*i*_ is less than 1.0) and 167 high wind speed measuring points (wind speed ratio *R*_*i*_ is greater than 1.0). Therefore, the distribution map of the corresponding simulation results is first given (Figure 6).

From the distribution results of the index *q*, there is a certain error between different working conditions of the SRAMS model, but the error is mainly concentrated in the low wind speed area, that is, the area where the wind speed ratio *R*_*i*_ is less than 1.0. On the other hand, it performs well in the high wind speed area, that is, the area where the wind speed ratio *R*_*i*_ is greater than 1.0. This is mainly due to the fact that the SRNS model cannot accurately simulate the flow separation phenomenon in the wake area of the building, which makes it poorly simulated in the low wind speed area. The LES condition performs well in both low wind speed and high wind speed regions.

In the CFD numerical simulation, the dimensions of all models are kept consistent with the wind tunnel test. The size of the computational domain is 15H (length) × 10H (width) × 6H (height) (as shown in Figure 7), and the blockage rate of the CFD numerical simulation is less than 3%, which meets the requirements of computational wind engineering and does not need to be revised. The structured grid is used for division, and the grid is refined at the building wall. The grid height of the first floor is 0.0002 meters. According to the preliminary simulation results, the *y* value of the building surface is about 30, the grid growth rate is set to 1.1, and the total number of grids for all working conditions is 7 × 10^7^ ~ 9 × 10^7^.

This paper takes the square enclosed layout as an example to verify the grid independence. First, a set of basic grids is established. The height of the first layer grid is 0.0002 meters, the grid growth rate is set to 1.1, and the total number of grids is about 7 million. Secondly, another two sets of grids of different sizes are distributed and established. The grid size of the first layer of the sparse grid is 0.0004 meters, the grid growth rate is 1.1, and the total number of grids is about 4 million. The mesh size of the first layer of the refined mesh is 0.0001 meters, the mesh growth rate is 1.1, and the total number of meshes is about 11 million. The corresponding grid size comparison chart is shown in Figure 8. Furthermore, different grids are used to simulate the pedestrian wind environment, and the calculation results of 26 different measuring points are obtained. The corresponding results are compared in Figure 9.

The article "Application of Mathematical Methods Based on Improved Fuzzy Computing in Building and Urban Design in the Environment of Industry 4.0" was published in 2022. Journal: Comput Intell Neurosci.

It can be clearly found that there is a significant difference in the calculation results between the sparse grid and the basic grid, while the difference between the refined grid and the basic grid is very small. This is enough to show that using the basic grid for simulation can not only ensure the calculation accuracy but also ensure that the computing resources are consumed as little as possible, so all the calculation case grids in this chapter are divided according to the basic grid method.

It can be seen from the foregoing that the self-sustainability of the wind speed must be ensured first before CFD numerical simulation is carried out. In this paper, the self-sustainability of wind speed is achieved by modifying the wall function and roughness parameters. The relevant simulation results are shown in Figure 10. The results show that the velocity profiles of the inlet and outlet are relatively consistent and have good self-sustainability in the verification results of the empty wind field.

When evaluating the pedestrian wind environment around a building, the wind speed ratio *R*_*i*_ is often used for analysis, and its related definition is as follows:

(9) $$\begin{array}{c} R_{i}=\frac{V_{i}}{V_{0}}, \end{array}$$

where *V*_*i*_ is the wind speed at the pedestrian height at the measuring point around the building (this paper is 2 meters above the ground), and *V*_0_ is the wind speed at the entrance pedestrian height when there is no building.

In order to quantitatively analyze the impact of building shape and layout on the pedestrian wind environment of high-rise buildings, this paper uses the maximum wind speed ratio *R*_max_ and the normalized accelerated area ratio *A*^*∗*^ ^*∗*^ to evaluate the wind environment of the building group. The relevant definitions are as follows:

(10) $$\begin{array}{c} R_{\max,\theta }=\max\left(R_{i,\theta }\right),\\ A_{R,\theta }^{*}=\frac{A_{R,\theta }}{A_{T}},\\ R_{\max}=\max\left(R_{\max,\theta }\right),\\ R_{\min}=\min\left(R_{\max,\theta }\right),\\ A_{\max^{*}}=\max\left(A_{R,\theta }^{*}\right),\\ A_{\min^{*}}=\min\left(A_{R,\theta }^{*}\right),\\ A_{R,\text{arg}}^{*}=\frac{1}{N}\sum A_{R,\theta }^{*}, \end{array}$$

where *R*_i,*θ*_ is the wind speed ratio in the evaluation area when the wind direction angle is *θ*, and *A*_*T*_ is the area of the evaluation area. According to the distribution of measuring points, the size of this area is 900 × 900mm^2^. *θ*_*Rθ*_ is the size of the area where the wind direction angle is *θ* and the wind speed ratio in the area is greater than R (Figure 11).

The article "Application of Mathematical Methods Based on Improved Fuzzy Computing in Building and Urban Design in the Environment of Industry 4.0" was published in 2022. Journal: Comput Intell Neurosci.

It can be known from the previous definition that the size of the *R* value in *A*_*R*,*θ*_ should be a value greater than 1.0. Regarding the specific value of *R*, in the absence of meteorological statistics, in order to meet the comfort of the wind environment, the wind speed ratio of the dominant wind direction should not be greater than. Therefore, when conducting research in this paper, *R*_*i*_=1.2 is selected for research; that is, the magnitude of *A*_*R*,*θ*_ is calculated for wind environment assessment.

## 4. Application of Mathematical Methods Based on Improved Fuzzy Computing in Building and Urban Design in the Environment of Industry 4.0

The intelligent model covers the structure and related facilities of the building in all aspects of design, construction, and operation management. It is necessary to simplify the BIM model for different applications, filter the geometric and semantic data irrelevant to the visual analysis, and extract the key elements required for the approval of building spacing. The specific process of extracting key elements is shown in Figure 12.

On the basis of the above research, the effect of the model proposed in this paper is verified. The model in this paper mainly assists the architectural structure design and human experience in urban architectural design. Therefore, this paper combines the simulation test to evaluate the effect of architectural and urban design and evaluates the architectural experience. The results shown in Tables 1 and 2 are obtained.

From the above research, we can see that the urban design intelligent system proposed in this paper meets the needs of urban design in the environment of Industry 4.0.

## 5. Conclusion

The urban building has a significant impact on the city block in which it is located. In its sheer size and population alone, it is of obvious importance to the concentration of urban blocks, to pedestrians on the street, and to the streetscape itself. Moreover, these can be attributed to the environmental relationship of tall buildings, which must be the subject of effective urban design in a certain location. At this level, the development of urban building can be controlled by planners through local planning. Due to their relative volume and height, high-rise buildings have a great impact on the existing surrounding environment and the scale of the city. Whether standalone or blended into an urban environment, the larger the building's mass, the greater the impact. This paper combines the mathematical method of improving fuzzy calculation to construct the intelligent building and urban design system and improves the effect of urban architectural design through the intelligent model. The simulation results show that the urban design intelligent system proposed in this paper meets the needs of urban design in the environment of Industry 4.0.

The article "Application of Mathematical Methods Based on Improved Fuzzy Computing in Building and Urban Design in the Environment of Industry 4.0" was published in 2022. Journal: Comput Intell Neurosci.

## Figures and Tables

**Figure 1:** Basic model parameters. (a) Model size. (b) Average wind speed profile and turbulence intensity. (c) Distribution map of measuring points.

**Figure 2:** Computational domain and boundary condition settings (square).

**Figure 3:** Schematic diagram of grid distribution (square).

**Figure 4:** Grid independence analysis (square). (a) Basic network. (b) Encrypted Network. (c) Sparse network.

**Figure 5:** Comparison of inlet and outlet wind speed profiles under different conditions. (a) Unadjusted wind profile comparison. (b) Adjusted wind profile comparison.

**Figure 6:** Distribution results of evaluation index q value under different working conditions. (a) Standard K-*ε* model. (b) RNG K-*ε* model. (c) Realizable K-*ε* model. (d) Standard K-*ε* model. (e) SST K-*ε* model. (f) ARFE method. (g) CDRFG method.

**Figure 7:** Computational domain and boundary condition settings (building group).

**Figure 8:** Grid independence analysis (building group). (a) Global network. (b) Sparse network. (c) Base network. (d) Encryption network.

**Figure 9:** Comparison of wind speeds at different measuring points (buildings).

**Figure 10:** Comparison of inlet and outlet wind speed profiles under different working conditions (building group).

**Figure 11:** Schematic diagram of the calculation of *θ*_*R*,*θ*_.

**Figure 12:** Application process of the mathematical method based on improved fuzzy calculation in building and urban design.

**Table 1:** Evaluation of architectural and urban design effects.

Number	City design	Number	City design	Number	City design
1	77.73	26	74.89	51	72.16
2	74.16	27	80.02	52	77.88
3	70.21	28	75.51	53	76.07
4	74.21	29	75.06	54	81.58
5	80.27	30	73.25	55	83.74
6	76.40	31	73.41	56	74.14
7	78.11	32	69.83	57	82.05
8	81.21	33	73.41	58	77.35
9	79.30	34	83.55	59	81.83
10	71.06	35	83.59	60	78.62
11	76.57	36	74.58	61	74.05
12	83.50	37	72.94	62	83.96
13	72.94	38	70.72	63	81.90
14	70.08	39	69.63	64	81.18
15	69.94	40	78.15	65	77.22
16	75.85	41	71.83	66	80.56
17	75.67	42	77.15	67	78.62
18	82.61	43	82.67	68	73.14
19	82.39	44	80.56	69	79.49
20	78.42	45	79.20	70	79.93
21	72.81	46	74.98	71	70.61
22	80.63	47	71.22	72	80.45
23	70.59	48	73.28	73	71.19
24	83.27	49	77.99	74	71.76
25	77.91	50	82.50	75	76.45

The article "Application of Mathematical Methods Based on Improved Fuzzy Computing in Building and Urban Design in the Environment of Industry 4.0" was published in 2022. Journal: Comput Intell Neurosci.

**Table 2:** User experience evaluation of urban design.

Number	User experience	Number	User experience	Number	User experience
1	84.17	26	86.03	51	79.97
2	80.32	27	77.55	52	84.71
3	85.38	28	74.59	53	83.20
4	77.41	29	76.95	54	79.83
5	79.55	30	76.04	55	86.98
6	78.61	31	76.00	56	78.19
7	74.66	32	77.55	57	82.80
8	79.65	33	79.73	58	74.43
9	74.12	34	79.06	59	86.00
10	79.25	35	85.93	60	84.08
11	73.26	36	75.26	61	76.00
12	85.37	37	83.04	62	77.24
13	74.69	38	83.38	63	73.88
14	77.81	39	73.57	64	84.99
15	74.33	40	82.82	65	74.01
16	83.27	41	77.29	66	83.80
17	85.23	42	81.82	67	83.52
18	84.34	43	86.01	68	76.88
19	73.82	44	74.03	69	85.64
20	80.35	45	76.39	70	83.58
21	82.51	46	73.88	71	86.91
22	76.22	47	83.24	72	82.34
23	82.53	48	78.80	73	73.42
24	73.25	49	82.78	74	81.34
25	84.09	50	74.67	75	86.60

## Data Availability

The labeled dataset used to support the findings of this study is available from the corresponding author upon request.
